The article "Study on the Nursing Effect of Diabetes Health Education Nursing Methods Applied to Diabetes Patients in the Endocrinology Department" was retracted in 2023. Reasons: signs of a paper mill; suspected computer-generated content; unreliable results or conclusions; lack of ethics approval or compliance.

# Study on the Nursing Effect of Diabetes Health Education Nursing Methods Applied to Diabetes Patients in the Endocrinology Department

**DOI:** 10.1155/2022/3363096

**Published:** 2022-01-04

**Authors:** Jianhua Wang, Yanan Zhao, Fei Xie

**Affiliations:** Qingdao Municipal Hospital, Qingdao 266000, China

## Abstract

The aim of this study was to explore the nursing effect of diabetes education and nursing methods applied to diabetic patients in the endocrinology department. From October 2019 to October 2020, 90 patients with diabetes who were admitted to the Department of Endocrinology in our hospital were selected as the research objects, and the medical records of all patients were retrospectively analyzed. The patients were randomly divided into two groups, 45 patients who were given regular care as the control group and 45 patients who were given the diabetes health education care model as the experimental group. Routine care was given to patients in the routine group; that is, we paid attention to the patients' diet, medication, and blood glucose levels. The experimental group patients were given diabetes health education guidance. The nursing effect, blood sugar level, disease awareness level, occurrence of complications, and compliance of the two groups of patients were evaluated. In this study, diabetes health education was given to the experimental group of patients. The conditions of this group of patients were significantly better than those of the basic group using conventional nursing methods. Therefore, the application of diabetes health education is very effective. The recovery from the disease has positive significance.

## 1. Introduction

Diabetes is a very common disease in the entire clinic. It belongs to the endocrine system disease. It not only has great harm but also the patient's organs and systems will suffer very serious damage, and sometimes, it may even cause it. Diabetic feet and diabetic kidneys, as well as various diseases such as chloasma of the fundus and peripheral audit damage, directly lead to a continuous decrease in the quality of life of patients [1–3]. In clinical medicine, there is no good method for the treatment of diabetes at this stage, but more attention is paid to the patient's comprehensive life intervention, which can effectively improve the prognosis and prevent the complications of diabetes. The treatment of diabetes is a long process, so it is very important to do a good job of health education during the treatment. Diabetes, as the most common chronic disease, has a very high clinical incidence. The patient's long-term high blood sugar state will cause blood vessels and organs to develop diseases, trigger a variety of complications, and threaten patients' life safety in severe cases. For diabetic patients, long-term medications to control blood sugar are needed, but adverse emotions will also affect the treatment during the treatment of the patient's disease, which will reduce the patient's treatment compliance. If the patient's knowledge of the disease is poor, it will also reduce their treatment compliance [4–6].

The article "Study on the Nursing Effect of Diabetes Health Education Nursing Methods Applied to Diabetes Patients in the Endocrinology Department" was retracted in 2023. Reasons: signs of a paper mill; suspected computer-generated content; unreliable results or conclusions; lack of ethics approval or compliance.

## 2. Materials and Methods

General information: 90 diabetic patients admitted to our hospital's Department of Endocrinology from October 2019 to October 2020 were selected as the research objects, and the medical records of all patients were retrospectively analyzed. The patients were randomly divided into two groups, 45 patients who were given regular care as the control group 45 patients who were given diabetes health education and nursing mode as the experimental group, and the general data such as gender and age of the two groups were compared. There was no statistical difference.

Routine care was given to patients in the routine group; that is, we paid attention to the patient's diet, medication, and blood glucose levels. The experimental group patients were given diabetes health education guidance, and the main operation methods are as follows: Firstly, a diabetes education and nursing research team is built. The director of the endocrinology department, professional diabetes-attending physicians, nursing physicians, head nurses, and key nurses in the department, combined with nutritionists and psychologists, jointly formed a diabetes healthcare research team in the hospital. Secondly, when the patient comes to the hospital for treatment, the nursing staff should enthusiastically and actively communicate with the patient and their family members about the patient's condition, fully grasp the patient's understanding of diabetes, life, eating habits, and physical conditions, and then, build an electronic account of the patient's condition. They should file and continue to improve in the future treatment process. At the same time, it is necessary for the attending physician in the undergraduate room to inform patients on how to control blood sugar so that patients can realize the importance of effective blood sugar control and then effectively control the development of their own disease and complications. Thirdly, during the patient's hospitalization, nursing staff should distribute diabetes health education brochures or leaflets to every patient and appropriately explain the pathogenesis, types, related complications, and correct methods of how to control blood sugar to patients. At the same time, the director of the endocrinology department should regularly organize patients to give lectures on the condition of “diabetes” so that patients can fully understand the correct methods of personal hygiene, diet, exercise, and medication after illness and promote patients in future treatment to eat healthy, exercise rationally, and use scientific medications so that blood sugar can be effectively controlled and patients' self-management ability can be improved so that the continued development of the disease can be controlled and the incidence of complications can be reduced. In addition, the nursing staff should also carry out appropriate education and publicity to the family members of the patients so that the family members can assist the patients in the control of the disease as much as possible and supervise the patients to carry out effective self-management. Finally, nursing staff should patiently instruct patients when they are discharged from the hospital and at the same time, according to the conditions of different patients, formulate relevant care plans and instruct patients to come to the hospital for review on a regular basis. Nursing staff should conduct regular telephone follow-ups after the patients are discharged from the hospital, to grasp the patient's recovery and adjust the care plan in time for the patients' recovery so that the patients can get better care. The department should also set up a consultation hotline to provide convenience for patients' consultation after discharge. It can also establish a patients' WeChat group so that different patients can discuss their conditions together, share treatment experiences, and encourage each other. The nursing effect, blood sugar level, disease awareness level, occurrence of complications, and compliance of the two groups of patients were evaluated. SPSS 22.0 software was used to perform statistics on the data in the text, *t* and chi-square were regarded as test indicators, and *P* < 0.05 was regarded as statistically different.

The article "Study on the Nursing Effect of Diabetes Health Education Nursing Methods Applied to Diabetes Patients in the Endocrinology Department" was retracted in 2023. Reasons: signs of a paper mill; suspected computer-generated content; unreliable results or conclusions; lack of ethics approval or compliance.

## 3. Results

### 3.1. Comparison of General Information of the Two Groups of Patients

By comparing the general information of the two groups of patients, it was found that there was no significant statistical difference between the patients in terms of gender, age, and time of illness (*P* > 0.05). Table 1 shows the comparison of general information of the two groups of patients.

### 3.2. Comparison of Nursing Effects between the Two Groups of Patients

After comparing the nursing effect of the two groups of patients, it was found that the nursing effect of the experimental group was better and the total effective rate was higher. The difference between the two groups was statistically significant (*P* < 0.05).  Table 2 is a comparative analysis of the nursing effect of the two groups of patients.

### 3.3. Differences in Blood Glucose Levels and Disease Awareness between the Two Groups

After comparing the blood glucose levels and disease cognition levels of the two groups of patients, it was found that compared with the control group, the fasting blood glucose and the 2 h postmeal blood glucose levels of the experimental group were lower, and the difference was statistically significant. In addition, compared with the control group, the disease cognition level of the experimental group was significantly higher than that of the control group, and the difference was statistically significant (*P* < 0.05). Table 3 displays the comparison of blood glucose level and disease awareness level.

### 3.4. Comparison of Complications

Comparing the incidence of the two groups of patients, it was found that the complication rate in the experimental group was 6.7%, including 1 case of hypoglycemia and 2 cases of heart failure. The complication rate of the control group was 11%, including 2 cases of hypoglycemia. There were 2 cases of heart failure and 3 cases of angina pectoris. The difference between the two groups was statistically significant (*P* < 0.05).

### 3.5. Compliance Assessment of the Two Groups of Patients

The effective rate of treatment compliance assessment in the experimental group was 91.1%, which was significantly higher than the 75.6% in the control group (*P* < 0.05).  Table 4 shows the compliance assessment of the two groups of patients.

## 4. Conclusions

Diabetes patients have higher blood sugar, which is generally caused by autoimmune problems, obesity, environment, genetics, and other factors. Diabetes is caused by a variety of factors. The patients in this study all belong to type 2 diabetes, and diabetes can be controlled by taking medicine. According to related studies, it is difficult to achieve better curative effect if only relying on drugs to treat diabetes, but health education can improve the treatment effect of diabetes. Medical staff should implement health education for patients with diabetes, which can greatly improve patients' compliance with treatment [7, 8].

Nursing staff can use various forms to carry out health education. Nursing staff can analyze the patient's condition in detail and formulate a targeted education program based on the patient's condition. The patient's awareness of diabetes can be improved through demonstration, training, and seminars. The content of health education includes blood glucose testing methods, the significance of blood glucose control, and the normal range of blood glucose; the mechanism, symptoms, prognosis, and types of diabetes; methods, goals, and meanings of diet control; the amount of exercise during exercise, the choice of exercise time, etc; the impact of negative emotions on diseases and how to control negative emotions; side effects, indications, dosages, and time of administration of hypoglycemic drugs; and use, storage, injection methods and dosages of insulin. Through health education, patients can actively cooperate with the nursing staff and scientifically control their own behavior and diet, thereby gradually improving the treatment effect. Through this research, we know that the application of diabetes health education in endocrine patients can gradually increase the patient's treatment compliance and improve the patient's diet, behavior, and psychological status, which has a positive significance in improving the treatment effect [9, 10].

The article "Study on the Nursing Effect of Diabetes Health Education Nursing Methods Applied to Diabetes Patients in the Endocrinology Department" was retracted in 2023. Reasons: signs of a paper mill; suspected computer-generated content; unreliable results or conclusions; lack of ethics approval or compliance.

Diabetes is a metabolic disease. Most diabetic patients are accompanied by endocrine disorders. If not intervened in time, it is likely to lead to metabolic disorders, vascular disease, and serious development of the disease and can even threaten the lives of patients. Relevant studies have shown that endocrine disorders in diabetic patients are mostly related to living habits, work habits, and eating habits. Patients do not have a clear understanding of their own diseases and will not exercise self-control in their daily lives, resulting in poor treatment and prognosis. Therefore, in order to better ensure the treatment effect of diabetic patients, it is necessary to pay attention to health education in clinical practice. Through scientific and effective health education, we should help patients correct their bad living habits and eating habits. At the same time, we should let patients realize the importance of taking medication on time, thereby improving patient compliance with medication and improving treatment effects. Therefore, it is of great significance to do a good job of health education in the endocrine care of diabetic patients [11].

Nursing staff can use various forms to carry out health education. Nursing staff can analyze the patient's condition in detail and formulate a targeted education program based on the patient's condition. The patient's awareness of diabetes can be improved through demonstration, training, and seminars. The content of health education includes blood glucose testing methods, the significance of blood glucose control, and the normal range of blood glucose; the mechanism, symptoms, prognosis, and types of diabetes; methods, goals, and meanings of diet control; the amount of exercise during exercise, the choice of exercise time, etc.; the impact of negative emotions on diseases and how to control negative emotions; side effects, indications, dosages, and time of administration of hypoglycemic drugs; and use, storage, injection methods and dosages of insulin. Through health education, patients can actively cooperate with the nursing staff and scientifically control their own behavior and diet, thereby gradually improving the treatment effect. Through this study, it is known that the application of diabetes health education in endocrine patients can gradually increase the patient's treatment compliance and improve the patient's diet, behavior, and psychological status, which has a positive significance in improving the treatment effect [12–14].

The article "Study on the Nursing Effect of Diabetes Health Education Nursing Methods Applied to Diabetes Patients in the Endocrinology Department" was retracted in 2023. Reasons: signs of a paper mill; suspected computer-generated content; unreliable results or conclusions; lack of ethics approval or compliance.

In this study, by comparing the general information of the two groups of patients, it was found that the patients had no significant statistical differences in gender, age, and time of illness (*P* > 0.05). After comparing the nursing effect of the two groups of patients, it was found that the nursing effect of the experimental group was better, and the total effective rate was higher [15–17]. The difference between the two groups was statistically significant (*P* < 0.05) [18–20]. By comparing the blood glucose levels and disease cognition levels of the two groups of patients, it was found that compared with the control group, the fasting blood glucose and the 2 h postmeal blood glucose levels of the experimental group were lower, and the difference was statistically significant. In addition, compared with the control group, the disease cognition level of the experimental group was significantly higher than that of the control group, and the difference was statistically significant (*P* < 0.05) [21, 22]. Comparing the incidence of the two groups of patients, it was found that the complication rate in the experimental group was 6.7%, including 1 case of hypoglycemia and 2 cases of heart failure. The complication rate of the control group was 11%, including 2 cases of hypoglycemia. There were 2 cases of heart failure and 3 cases of angina pectoris. The difference between the two groups was statistically significant (*P* < 0.05). The effective rate of treatment compliance assessment in the experimental group was 91.1%, which was significantly higher than the 75.6% in the control group (*P* < 0.05).

In summary, in this study, the experimental group of patients was given diabetes health education. The conditions of this group of patients were significantly better than those of the basic group of patients using conventional nursing methods. Therefore, the application of diabetes health education is extremely effective. Also, it has a positive significance for the recovery of the disease.

The article "Study on the Nursing Effect of Diabetes Health Education Nursing Methods Applied to Diabetes Patients in the Endocrinology Department" was retracted in 2023. Reasons: signs of a paper mill; suspected computer-generated content; unreliable results or conclusions; lack of ethics approval or compliance.

## Figures and Tables

**Table 1:** Comparison of general information of the two groups of patients.

	Control group (*n* = 45)	Test group (*n* = 45)	T value	*P* value
Gender/male	21	23	1.56	0.08
Age	48.98 ± 10.36	46.58 ± 9.87	1.29	0.28
Sick time/year	5.6 ± 3.5	5.8 ± 3.1	0.65	0.58

**Table 2:** Comparative analysis of the nursing effect of the two groups of patients (%).

Group	Markedly effective	Effective	Invalid	Total effective rate
Test group (*n* = 45)	22	18	5	88.8%
Control group (*n* = 45)	16	17	12	73.3%
X2	—	—	—	8.95
*P* value	—	—	—	0.02

**Table 3:** Comparison of blood glucose level and disease awareness level (*x* ± *s*).

Group	Fasting blood glucose (mmol/L)	2 h blood glucose after meal (mmol/L)	Disease awareness level (points)
Test group (*n* = 45)	6.53 ± 2.56	8.16 ± 3.25	95.68 ± 4.58
Control group (*n* = 45)	9.56 ± 2.64	10.26 ± 2.68	85.36 ± 3.56
T value	5.48	5.64	12.68
*P* value	≤0.01	0.01	≤0.01

**Table 4:** Compliance assessment of the two groups of patients.

Group	High compliance	Moderate compliance	Poor compliance	Evaluation efficiency
Test group (*n* = 45)	30	11	4	91.1%
Control group (*n* = 45)	26	8	11	75.6%
X^2^	—	—	—	6.54
*P* value	—	—	—	0.01

## Data Availability

The simulation experiment data used to support the findings of this study are available from the corresponding author upon request.
